# Catheter Directed Thrombolysis in the Treatment of Acute Pulmonary Embolism: Early Hemodynamic Recovery and Improvement in Prognosis

**DOI:** 10.1155/2022/4846279

**Published:** 2022-03-24

**Authors:** Qinglong Guan, Xiaofei Wang, Chenglong Liu, Yuan Gao, Haibo Chen, Gang Li

**Affiliations:** ^1^Department of Vascular Surgery, The Second Affiliated Hospital of Shandong First Medical University, Taian 271000, China; ^2^Medical Laboratory, The Second Affiliated Hospital of Shandong First Medical University, Taian 271000, China; ^3^Department of Radiology, The Second Affiliated Hospital of Shandong First Medical University, Taian 271000, China

## Abstract

**Aim:**

In this study, we aimed to investigate the efficacy of catheter directed thrombolysis (CDT) and peripheral intravenous thrombolysis (PIT) in the treatment of patients with acute pulmonary embolism (APE) and assess its effect on the prognosis of patients.

**Methods:**

We recruited 74 patients with APE, who were assigned to CDT and PIT groups, according to the treatments received by them. The arterial partial pressure of oxygen (PaO_2_), partial pressure of carbon dioxide (Pa CO_2_), pulmonary artery pressure (PAP), pulmonary artery obstruction index (PAOI), thrombus volume, pain score, and therapeutic benefits were compared between the two groups before and after treatment, and the factors affecting patient prognoses were also analyzed.

**Results:**

Using the clinical data before treatment as the baseline, it was found that changes in indicators of plasma, thrombus volume, and pain scores were significantly better in the CDT group than in the PIT group after treatment. The total effective rate of CDT was higher than that of PIT in the treatment of APE. The mean follow-up time for both the CDT and PIT groups was 41.08 ± 9.12 months, and the total mortality rate was 14.8% and 31%, respectively. The logistic regression analysis revealed the significant impacts of previous incidences of pulmonary embolism (PE), concurrent deep vein thrombosis (DVT), and pulmonary arterial hypertension (PAH) on the occurrence and progression of APE, and these factors were subsequently identified as risk factors for APE using Kaplan–Meier survival analysis. Observations from PAE onset to the end of follow-up revealed that there was a difference in survival rates between the CDT and PIT groups.

**Conclusions:**

Taken together, CDT is an effective treatment strategy for APE and can provide effective symptomatic relief. In addition, the previous incidences of PE, concurrent DVT, and PAH are important risk factors that affect the survival rates of patients with APE.

## 1. Introduction

Acute pulmonary embolism (APE) is a clinical syndrome that is a result of the obstruction of a pulmonary artery or its branches by a variety of endogenous or exogenous emboli. In the United States of America (USA), the incidence of APE is as high as 40-50 cases per 100,000 people per year, with a total of over 900,000 individuals affected by this disease [1]. Moreover, APE is also a common cause of sudden and unexpected deaths in China. Misdirected or untimely treatment of APE leads to a mortality rate of approximately 50%–80%. However, this mortality rate can be reduced to 2%–8% [2]. As APE is often misdiagnosed and is currently under-recognized in all levels of hospitals in China, it is critical to accurately diagnose APE and evaluate its severity using current laboratory biological markers, including plasma D-dimer, brain natriuretic peptide (BNP), and PE scoring index (PESI) [3]. The current treatment strategies for APE include anticoagulation alone, peripheral intravenous thrombolysis (PIT), and catheter directed thrombolysis (CDT). The use of anticoagulation alone is associated with right ventricular (RV) dilatation, which has a high mortality rate [4]. In patients with severe APE receiving PIT, although hemodynamic disturbances are reduced, the risk of bleeding is increased. Currently, commonly used thrombolytic drugs include urokinase (a type of first-generation drug) and recombinant human tissue-type plasminogen kinase derivatives (Reteplase) (r-PA, a type of third-generation drug). Studies have shown that approximately 7% of the patients with acute bleeding and 4% of the patients with systemic thrombolysis require transfusion after receiving thrombolytic drugs [5]. In the CDT treatment, the site of venous thrombosis is identified under pulmonary arteriography, a catheter is inserted into the main trunk and branches of the involved pulmonary artery, and thrombolysis is performed; this is a highly effective treatment approach for APE [6] and can minimize complications. CDT can rapidly decrease RV strain in patients within 48 h of their admission [7] and reduce the volume of thrombi in their pulmonary arteries. Therefore, effective diagnosis and selection of an appropriate treatment strategy can reduce the mortality rates of patients with APE. In this study, the clinical efficacy, safety, risk factors, and improvement of prognosis exhibited by PIT and CDT approaches were evaluated by retrospectively analyzing 74 patients with APE. The relevant guidelines only outline the details on the usage of urokinase in the treatment of APE, without specific guidance on the dose, timing of administration, and mode of administration of r-PA; furthermore, there is a lack of targeted guidance regarding the treatment of APE. Therefore, this study provides a theoretical basis for the treatment of APE in terms of treatment choices and drug selection, thus guiding clinicians in choosing the best treatment or strategy to improve the efficacy of treatment for patients with APE.

## 2. Materials and Methods

### 2.1. Patient Detail

In this study, 74 patients diagnosed with APE at the Second Affiliated Hospital of Shandong First Medical University between January 2015 and January 2017 were recruited. The diagnostic criteria used were in accordance with those outlined by the Chinese Expert Consensus on the Diagnosis and Management of Acute Pulmonary Embolism and the 2014 European Society of Cardiology Guidelines on the Diagnosis and Treatment of Acute Pulmonary Thromboembolism [8, 9]. Inclusion criteria for this study were as follows: (i) pulmonary arteriography showing embolism in more than two lobes or seven lung segments, confirmed through pulmonary CT angiography and color Doppler ultrasound; (ii) cardiac function and laboratory tests showing right ventricle (RV) insufficiency and myocardial injury, but no significant hemodynamic changes; and (iii) no contraindications to anticoagulation or thrombolysis. The exclusion criteria were as follows: (i) patients with a high-risk classification for APE (defined as syncope, systemic arterial hypotension, cardiogenic shock, or cardiac arrest and resuscitation); (ii) patients with contraindications to thrombolysis (stroke or transient ischemic attack; recent active bleeding from major organs); and (iii) patients with moderate to severe chronic obstructive pulmonary disease (COPD), acute coronary syndrome (ACS), or cardiac insufficiency. The patients were informed of the risks associated with the procedures, and the protocol was determined after the principles of treatment were discussed with the patient or patient's family. The patients were assigned to PIT and CDT groups according to treatment strategy used, with 37 patients in each group. The study was approved by the Ethics Committee of the Second Affiliated Hospital of Shandong First Medical University. The details are provided in Table 1.

### 2.2. Methods

Patients in both the CDT and PIT groups were routinely administered 0.1 mL/kg of low molecular heparin calcium injections (Kunming Jida Pharmaceutical Co., Ltd., Yunnan, China, SFDA approval number: H20053198, specification: 0.6 mL) subcutaneously. Patients in the CDT group were administered r-PA through the dorsal vein of the foot at an injection standard of 9 mg/dose +0.9% NS (total dose = 100 ml, 6 h of intravenous drip), which was followed by another similar dose after 12 hours. Patients in the CDT group were administered interventional thrombolytic therapy. Specifically, a 5F catheter sheath was inserted through the femoral vein on the healthy side of a lower limb (if there was a lower limb vein thrombosis on the affected side); a 5F pigtail catheter was inserted; a pulmonary arteriogram was used to detect the extent, size, shape, and location of the thrombus in the pulmonary artery; and a catheter was inserted into the pulmonary artery to perform thrombolysis. The r-PA injection (approximately 9 mg/dose +0.9% NS, total volume = 50 mL) was then administered 5 minutes after the thrombolytic catheter was placed in the pulmonary artery. After 24 h of this procedure, r-PA was transfused for 6 hours at the same dose as the previous one. Changes in coagulation Indicators were monitored, and a catheterization was performed 3 days after the procedure to observe the effect of thrombolysis.

### 2.3. Observational Indicators and Efficacy Assessment Criteria

Laboratory tests included measurement and comparison of plasma D-dimer levels and arterial blood gases before and after treatment between the two groups; partial pressure of carbon dioxide (Pa CO_2_), arterial partial pressure of oxygen (Pa O2), and pulmonary artery pressure (PAP) were measured using an arterial blood-gas analyzer.

The volume of pulmonary artery obstruction was calculated using chest CTPA auxiliary analysis software, and the difference in volumes of obstruction before and after thrombolysis was measured; this was the reduced volume of the embolism. The pulmonary artery obstruction index (PAOI) was calculated based on the CTPA results and using the Mastora method [10].

Changes in relevant indicators, such as D-dimer levels, PAOI, thrombus volume, and pain score, before and after treatment were compared between the two groups. The criteria used to assess the clinical efficacy of the two treatment approaches were as follows: (i) marked effective: complete remission of symptoms, complete restoration of vascular flow, with no complications; (ii) effective: partial remission of symptoms, partial restoration of blood flow, with few complications; and (iii) ineffective: no remission of symptoms, with significant pulmonary thrombosis.

### 2.4. Statistical Analysis

All data from this clinical study were analyzed using the SPSS 22.0 (IBM Corporation, Armonk, NY, USA). The enumeration data were expressed as cases (%), and the *χ*^2^ or Mann–Whitney *U* test were used for cohort comparisons. The measurement data were expressed as $\overset{¯}{\text{X}}\pm \text{S}$, and the analysis was performed using the *t*-test. Unless otherwise stated, *P* < 0.05 was considered statistically significant during all analyses.

## 3. Results

### 3.1. Comparison of Changes in Vital Signs between the CDT and PIT Groups

After treatment, D-dimer levels decreased to the normal range in the CDT group and were significantly lower than that in the PIT group, with a significant difference (*P* < 0.01); in addition, the means of PaCO_2_, PAP, and PAOI in the CDT group were significantly lower than those in the PIT group, and PaO_2_ was significantly higher in the CDT group than that in the PIT group (*P* < 0.01), as shown in Table 2.

The difference in thrombus volume and pain score between the CDT and PIT groups before treatment was not statistically significant (*P* > 0.05). At three days and one week after treatment, the thrombus volume decreased significantly (*P* < 0.01) in both groups, with a greater decrease in the CDT group, as shown in Table 3.

### 3.2. Analysis of Efficacy in the Two Groups

Patients in both groups were administered thrombolytic treatment using different strategies. Based on our results, the clinical benefit obtained by the patients in the CDT group, with a total effective rate of 97.2%, was higher than that obtained by the patients in the PIT group, with a total effective rate of 81.0%, as shown in Table 4 and the Figure 1.

### 3.3. The Effect of Multiple Factors on the Occurrence and Progression of APE

We constructed a multivariate logistic regression equation for concurrent DVT, previous incidences of PE, previous incidences of VTE, and PAH in patients with APE. The results revealed that higher incidences of concurrent DVT correlated with increased risk of APE progression (OR = 5.89, 95%CI = 1.15–30.02, *P* = 0.03). The previous incidence of PE correlated with an increased risk of recurrent APE (OR = 4.40, 95%CI = 1.16–16.68, *P* = 0.02). PAH was significantly associated with an increased risk of APE onset (OR = 6.22, 95%CI = 1.45–26.59, *P* = 0.01). The previous incidence of VTE was not correlated with an increased risk of APE onset (OR = 1.99, 95%CI = 0.51–7.78, *P* = 0.31), as shown in Table 5.

### 3.4. Comparison of the Survival Curves of Patients in the Two Groups

The above data reveal the impact of previous incidences of PE, concurrent DVT, and PAH on the progression of APE and prognoses of patients with APE. The survival status of patients with APE was assessed in this study, with a mean follow-up duration of 41.08 ± 9.12 months (median, 24.6 months) in both the CDT and PIT groups. The total mortality rate was 14.8% and 31% in the CDT and PIT groups, respectively (*P* = 0.01). Kaplan–Meier survival curves for patients with previous incidences of PE, concurrent DVT, and PAH were analyzed during APE follow-up, and the log-rank values were found to be 2.96, 12.75, and 4.35 with *P* values of 0.08, 0.01, and 0.03, respectively, indicating that the survival rates were significantly higher in the CDT group than in the PIT group. Moreover, the survival rate curve in the CDT group showed an exponential increase from 0 to 2000 days, while the survival rate curve in the PIT group showed a slow increase from 0 to 2000 days. These results indicated that the CDT approach showed better efficacy than did the PIT approach in the treatment of patients with APE, as shown in Figure 2.

## 4. Discussion

PE is a pulmonary circulation disorder that is caused by the obstruction of the main pulmonary artery or its branches by thrombi or other material dislodged from limb veins; it is mostly associated with the formation and dislodgement of DVT [11]. PE can lead to a series of pathophysiological changes in the patients' body, and the typical symptoms include hemoptysis, polypnea [12], dyspnea, acute right heart failure [13]_,_ and even death. If PE is not treated in a timely manner effectively, it may lead to death. Recent advances in therapeutics have led to the adoption of a comprehensive and minimally invasive treatment approach for APE [14]. CDT reduces the size of emboli in the main pulmonary artery through fragmentation, allowing them to enter the distal branches of the pulmonary artery, thereby opening up the main pulmonary artery and improving RV function. Another study have shown that CDT has a significant advantage over anticoagulation and PIT alone in the treatment of APE [15]. Overall, CDT relieves relevant symptoms of APE patients, maintains the stability of patients' vital signs after surgery, and improves the prognosis.

CDT administration is achieved by infusing thrombolytic drugs into the pulmonary artery of patients. The third-generation thrombolytic drug rPA converts plasminogen into active fibrinoclase to degrade fibrin in thrombi and exerts a thrombolytic effect.

Currently, the clinical application of r-PA in thrombolytic treatment of acute myocardial infarction has demonstrated satisfactory clinical outcomes, but the recommended dosage and optimal administration protocols in the treatment of APE have not been explored. However, increasing the dose of r-PA that is perfused into the pulmonary artery through interventional treatments can increase the local drug concentration and thus enhance the thrombolytic effect. Studies have shown that elevated D-dimer levels indicate hypercoagulability and secondary hyperfibrinolysis [16, 17]. Therefore, the D-dimer levels are important for the diagnosis and assessment of outcomes and patients' prognoses in thrombotic diseases and are often used as a marker of the severity of APE, with reduced levels indicating an improvement in the patients' condition [18]. In another study [19], arterial blood gas analyses revealed hypoxemia in PE patients, with abnormal blood gas status and increased differences in alveolar-arterial partial pressures. Herein, we found that patients in the CDT group exhibited greater improvement in Pa CO_2_, Pa O_2_, and PAP levels than did the patients in the PIT group, suggesting that CDT had a facilitating effect on the recovery of arterial blood gas in patients with APE, relieved pulmonary artery obstruction symptoms, promoted the patients' intrapulmonary air-blood exchange, corrected hyperventilation, reduced the occurrence of PAH, and improved the patients' prognosis. At different time points before and after CDT treatment, the patients' pain scores and thrombus volume were found to be significantly reduced, indicating a significant improvement in the patients' typical symptoms.

The main feature of CDT is that it restores blood flow to the main pulmonary artery in a short period of time, which leads to a protective effect on the pulmonary artery and the right atrium and ventricle and reduces the occurrence of related complications later in life. The multivariate logistic regression equation constructed in this study helped reveal that higher incidences of concurrent DVT, previous incidences of PE, and PAH correlated with increased risk of APE recurrence. In the case of DVT, due to the patients' previous history of lower limb venous thrombosis, APE could occur again after thrombus dislodgement because of external triggers, such as trauma, surgery, and vascular injury, or due to genetic factors affecting thrombus recurrence. In patients with previous incidences of PE or PAH, the poor outcomes of previous anticoagulation therapies could lead to a reduction in pulmonary reserve capacity and a compensatory increase in RV function. Therefore, when venous thrombosis is dislodged, reaggravation of pulmonary embolism is possible. In the present study, the efficacy of both treatments (CDT and PIT) was analyzed, and there was a statistically significant difference in the total effective rate between the CDT and PIT groups. Based on the clinical data of the two groups obtained herein, we found that the patients' prognosis was influenced by previous incidences of PE, concurrent DVT, and PAH and that the prognosis of patients receiving the CDT treatment was better than that of patients receiving the PIT treatment; these results are consistent with the results of previous studies [20]. CDT treatment is an invasive procedure, and the patients receiving CDT treatment bear a higher risk of complications and accidents than those receiving PIT treatment. However, CDT has been reported to be effective in reducing the mortality rate during early thrombolysis in PE [5]. Nevertheless, there is no evidence linking early thrombolysis to patient death caused by heart failure at long-term follow-up, but early thrombolysis can indeed help prevent such complications.

In conclusion, CDT is a highly effective approach for the treatment of patients with APE. Taken together, CDT was found to stabilize the patients' vital signs and improve their prognoses. The findings of this study showed that CDT combined with r-PA administration rapidly improved the hemodynamic parameters, laboratory indicators, and prognoses of patients with APE. Therefore, CDT can be considered a firstline therapy for patients with APE.

## Figures and Tables

**Figure 1:** Imaging images. (a, b) CT angiography (CTA) images of the pulmonary artery showing a filling defect in the right pulmonary artery trunk and branches (arrows) before treatment. (c) Pulmonary arteriogram showing a filling defect in the right pulmonary artery trunk and branches. (d) Pulmonary arteriogram 48 h after treatment. (e) CTA image of the pulmonary artery showing the disappearance of the filling defect in the right pulmonary artery trunk and branches. (f) The patency of blood flow in the pulmonary artery.

**Figure 2:** Comparison of survival curves of two groups of patients with different diseases.

**Table 1:** General clinical baseline data for patients enrolled in the study.

Clinical data	Peripheral intravenous thrombolysis group (*n* = 37)	CDT group (*n* = 37)	*P*
Age	56.72 ± 11.15	56.91 ± 10.42	0.923
Gender (M:F)	17 : 20	22 : 15	0.354
Previous PE	10 (27.0%)	11 (29.7%)	1.000
Previous VTE	14 (37.8%)	18 (48.6%)	0.482
Past hospital visit history			
Trauma history	12 (32.4%)	14 (37.8%)	0.808
Hyperlipidemia	17 (45.9%)	21 (56.8%)	0.797
Cardiovascular disease (CAD)	14 (37.8%)	16 (43.2%)	0.813
Obesity (BMI >25 kg/m^2^)	12 (32.4%)	11 (29.7%)	1.000
Whether there is DVT during the onset	25 (67.6%)	17 (45.9%)	1.000
Troponin	20 (54.1%)	23 (62.2%)	0.638
Pulmonary arterial pressure (mmHg)	46.79 ± 6.33	42.44 ± 7.13	0.581

**Table 2:** Differences in D-dimer levels, Pa CO_2_, Pa O_2_, PAOI, and PAO_2_ between the CDT and PIT groups.

Groups	D-dimer down to normal range/H	PaCO_2_/mm Hg	PaO_2_/mmHg	PAP/mm Hg	PAOI
Peripheral intravenous thrombolysis group	36.63 ± 11.74	35.25 ± 5.07	64.75 ± 4.66	46.97 ± 9.70	7.95 ± 2.32
CDT group	13.20 ± 4.81	29.14 ± 7.08	70.46 ± 7.54	36.61 ± 7.63	5.10 ± 1.52
*T* values	−11.13	5.48	−4.85	4.99	7.70
*P* values	≤0.01	≤0.01	≤0.01	≤0.01	≤0.01

Note: *P* < 0.05 was considered statistically significant.

**Table 3:** Remission of symptoms before and after CDT and PIT treatment in patients with APE.

Groups	Thrombus volume (V/cm^3^)			VAS Pain score (points)		
	Preoperative	3 days after surgery	1 week after surgery	Preoperative	3 days after surgery	1 week after surgery
CDT group	0.85 ± 0.37	0.72 ± 0.30	0.62 ± 0.24	5.16 ± 2.39	3.05 ± 1.12	1.91 ± 0.82
Peripheral intravenous thrombolysis group	0.91 ± 0.39	0.86 ± 0.38	0.80 ± 0.37	5.45 ± 2.32	4.13 ± 1.58	2.56 ± 1.25
*T* values	1.01	2.06	3.16	0.56	3.19	3.04
*P* values	0.32	0.04	≤0.01	0.57	0.003	0.03

**Table 4:** Efficacy of CDT and PIT treatments in patients with APE.

Groups	Effective		Efficient		Invalid		Total efficiency	
	*N*	%	*N*	%	*N*	%	*N*	%
CDT group	28	75.6	8	21.6	1	2.7	36	97.2
Peripheral intravenous thrombolysis group	13	35.1	17	45.9	7	18.9	30	81.0
*X* ^2^ values							3.69 0.04	
*P* values								

**Table 5:** Construction of the multivariate logistic regression equation.

	B	S.E.	Wals	df	Sig.	Exp (B)	95% CI of Exp (B)	
							Lower limit	Upper limit
With or without DVT	1.77	.83	4.55	1	.033	5.89	1.15	30.02
Previous PE	1.48	.68	4.76	1	.029	4.40	1.16	16.68
Previous VTE	.69	.69	.99	1	.319	1.99	.51	7.78
With or without pulmonary hypertension	1.82	.74	6.09	1	.014	6.22	1.45	26.59
Constant	-3.18	.82	14.97	1	.000	.04		

## Data Availability

The data presented in the study may be made available from the corresponding author upon reasonable request.
